RETRACTED

# A Bioinformatics Approach for the Prediction of Immunogenic Properties and Structure of the SARS-COV-2 B.1.617.1 Variant Spike Protein

**DOI:** 10.1155/2021/7251119

**Published:** 2021-10-05

**Authors:** Vijay Kumar Srivastava, Sanket Kaushik, Gazal Bhargava, Ajay Jain, Juhi Saxena, Anupam Jyoti

**Affiliations:** ^1^Amity Institute of Biotechnology, Amity University Rajasthan, Amity Education Valley, Kant Kalwar, NH-11C, Jaipur-Delhi Highway, Jaipur, India; ^2^Faculty of Applied Sciences and Biotechnology, Shoolini University of Biotechnology and Management Sciences, Bajhol, Solan, Himachal Pradesh, India

## Abstract

**Background:**

B.1.617.1, a variant of severe acute respiratory syndrome coronavirus-2 (SARS-CoV-2) causing respiratory illness is responsible for the second wave of COVID-19 and associated with a high incidence of infectivity and mortality. To mitigate the B.1.617.1 variant of SARS-CoV-2, deciphering the protein structure and immunological responses by employing bioinformatics tools for data mining and analysis is pivotal.

**Objectives:**

Here, an in silico approach was employed for deciphering the structure and immune function of the subunit of spike (S) protein of SARS-CoV-2 B.1.617.1 variant.

**Methods:**

The partial amino acid sequence of SARS-CoV-2 B.1.617.1 variant S protein was analyzed, and its putative secondary and tertiary structure was predicted. Immunogenic analyses including B- and T-cell epitopes, interferon-gamma (IFN-*γ*) response, chemokine, and protective antigens for SARS-CoV 2 S proteins were predicted using appropriate tools.

**Results:**

B.1.617.1 variant S protein sequence was found to be highly stable and amphipathic. ABCpred and CTLpred analyses led to the identification of two potential antigenic B cell and T cell epitopes with starting amino acid positions at 60 and 82 (for B cell epitopes) and 54 and 98 (for T cell epitopes) having prediction scores > 0.8. Further, RAMPAGE tool was used for determining the allowed and disallowed regions of the three-dimensional predicted structure of SARS-CoV-2 B.1.617.1 variant S protein.

**Conclusion:**

Together, the in silico analysis revealed the predicted structure of partial S protein, immunogenic properties, and possible regions for S protein of SARS-CoV-2 and provides a valuable prelude for engineering the targeted vaccine or drug against B.1.617.1 variant of SARS-CoV-2.

## 1. Introduction

Coronaviruses (CoVs), belonging to the family Coronaviridae, are enveloped nonsegmented, single-stranded positive-sense RNA viruses and infect humans and various animals (bats, birds, camels, cats, dogs, and mice) [1]. Based on the genome sequence, CoVs have been further categorized into four genera, i.e., the alpha, beta, gamma, and delta [2]. Six different species of CoVs infecting humans, all belonging to betacoronavirus, have been identified, i.e., human coronavirus (HCoV) 229E, HCoV-OC43, SARS-CoV, HCoV-NL63, HCoV-HKU1, and Middle East respiratory syndrome coronavirus (MERS-CoV). Except for SARS-CoV and MERS-CoV, the other four viruses cause the common cold in immunocompromised subjects [3].

RETRACTED

In 2003, the SARS-CoV emerged in Guangdong province in South China, which causes severe acute respiratory syndrome [4]. In 2012, the Middle East respiratory syndrome (MERS) was first identified in Saudi Arabia infecting ~2500 of which more than 800 resulted in death and rapidly spread in 27 countries across the globe [5]. Both SARS-CoV and MERS-CoV are zoonotic, and in human, they infect the upper respiratory tract causing common cold as well as lower respiratory tract resulting in bronchitis, whooping cough, and pneumonia [4, 5], and till to date, there is no approved therapeutic molecule for the treatment.

In December 2019, a large number of cases with pneumonia were reported and epidemiologically linked with the seafood market in Wuhan in Hubei province in China [6]. The causative agent was identified as novel CoV using state-of-art next-generation sequencing technology of the specimen isolated from the patient. Further, it has been coined the name SARS-CoV-2 due to 87% sequence similarity with the two bat-derived SARS-like CoV strains (bat-SL-CoVZC45 and bat-SL-CoVZXC21) having single-stranded RNA genome with size from 29 to 30 Kb [7, 8]. On 11 February 2020, the World Health Organization (WHO) named COVID-19 for the new disease caused by SARS-CoV-2 (https://www.who.int/emergencies/diseases/novel-coronavirus-2019/technical-guidance/naming-the-coronavirus-disease-(covid-2019)-and-the-virus-that-causes-it). COVID-19 rapidly spread across Asia (India, Iran, Japan, Pakistan, Saudi Arabia, South Korea, and Turkey), Europe (France, Germany, Italy, Netherlands, Switzerland, and the UK), North America (Mexico and the USA), South America (Brazil, Chile, and Peru), Africa (Algeria, Egypt, Ghana, Nigeria, and South Africa), and Oceania (Australia, New Zealand, and French Polynesia) (https://covid19.who.int/). The menace remains unabated and is continuously ravaging in other parts of the world. As of September 16, 2021, globally, there have been 225,680,357 confirmed cases of COVID-19, including 4,644,740 deaths (https://covid19.who.int/). Human to human transmission of SARS-CoV-2 has been reported, and infected patients are diagnosed with fever, cough, fatigue, and difficulty breathing [9, 10].

SARS-CoV-2 genome encodes several nonstructural, structural, and accessory proteins [11]. There has been a global endeavour by the researchers to decipher the structural-functional relations of the important proteins of SARS-CoV-2, to get an insight into the mechanistic details of their binding targets on human cells [11–15]. The S protein on the virus interacts with the angiotensin-converting enzyme 2 (ACE2) receptor present over human cells led to the internalization of SARS-CoV-2 within the cells [16]. Mutations in the S protein have been reported to enhance the binding with ACE2 [17]. The therapeutic strategies to inhibit the host recognition, and attachment of host with the virus by targeting S protein could be an attractive paradigm for developing anti-SARS-CoV-2 drugs.

RETRACTED

The ongoing global spread of SARS-CoV-2 has led to the emergence of new strains with profound and stable mutations. Among these strains, B.1.617.1 lineage first identified in India and subsequently spread to the other parts of the world are characterized by mutations in S as well as other proteins. This lineage has been categorized as variants of interest by CDC, hence underscoring the importance of study in terms of physiochemical properties, immunogenic potential, and protein structure prediction.

Both patient/host response and virus-specific information are pivotal in the clinical management of the disease including diagnosis and therapeutics. Recognition of the pathogen key protein by host cells to induce the immune system is of paramount importance as this is helpful in the designing of the vaccine. Identifying key pathogenic protein using homology modeling, a state-of-the-art bioinformatics tool is a viable strategy for designing of vaccine and therapeutic molecule. Further, identification of the permissible and nonpermissible regions is critical for identifying the potential drug targets with therapeutic efficacy.

Here, the in silico approach was employed to decipher the structure and function of the partial S protein of SARS-CoV-2 B.1.617.1 variant S protein. The SWISS-MODEL and PyMOL were used for the analysis of the amino acid sequence of SARS-CoV-2 B.1.617.1 variant S protein, and the prediction of the putative secondary and tertiary structure. Further, the ABCpred, TCLpred, CHEMOpred, and Vaxijen servers were used for identifying the immunoepitopes in the B.1.617.1 variant S protein. The RAMPAGE tool was then used for deducing and analyzing the Ramachandran plot for predicting the permissible and nonpermissible regions of the three-dimensional (3 D) structure of the SARS-CoV-2 B.1.617.1 variant S protein.

## 2. Materials and Methods

### 2.1. Physiochemical Characterization

ProtParam tool (http://web.expasy.org/protparam/) on ExPASy server was used for determining the physicochemical properties, i.e., molecular weight (Mw), isoelectric point (pI), amino acid composition, extinction coefficient (EC), instability index (II), aliphatic index (AI), and grand average of hydropathicity (GRAVY) of QUX03874.1 S protein [18].

RETRACTED

### 2.2. In Silico Prediction of Immunogenic Properties

Online tools including ABCpred [19], CTLpred [20], CHEMOpred [21], and Vaxijen server [22] were used to predict B-cell epitopes, CTL epitopes, chemokines, and protective antigen, respectively. B-cell epitopes in B.1.617.1 variant S protein QUX03874.1 were predicted using ABCpred tool (http://www.imtech.res.in/raghava/abcpred/). The QUX03874.1 S protein was also screened for the presence of potential CTL epitopes using CTLPred online server (http://www.imtech.res.in/raghava/ctlpred/). Both ABCpred and CTLpred are based on machine learning techniques such as artificial neural network and support vector machine, and epitope prediction was performed by employing a fixed-length pattern for the identification of continuous B-cell and T-cell epitopes with the threshold for scoring was set at 0.8. A higher score was commensurate with a higher probability of the existing epitope. Further, the antigenicity of the peptides was predicted using VaxiJen v2.0 tool (http://www.ddg-pharmfac.net/vaxijen/VaxiJen/VaxiJen.html). Further, interferon-gamma (IFN-*γ*) response for predicted epitopes was evaluated using the IFNepitope (http://crdd.osdd.net/raghava/ifnepitope/index.php) [23]. For the prediction of chemokines, ChemoPred, a support vector machine-based approach (https://webs.iiitd.edu.in/raghava/chemopred/index.html) was used with default parameters.

### 2.3. Alignment of the Sequence

The primary S protein sequence from SARS-CoV-2 B.1.617.1 variant, QUX03874.1, was identified from the ExPASy database [24]. The BLASTP against the Protein Data Bank (PDB) was carried out to determine the protein template for the QUX03874.1 and subsequent prediction of the model. The search revealed an identical sequence from Homo sapiens viral protein (Human SARS coronavirus) with PDB entry 7KQE [25]. This sequence was then used for in silico modeling. ClustalW tool [26] was used for the equivalent sequence alignment with 7KQE as a template.

### 2.4. Structure Prediction and Validation

SWISS-MODEL, a fully automated server that creates protein structure homology modeling [27], was used to predict the 3D structure of QUX03874.1 (partial S protein) from SARS-CoV-2 B.1.617.1 variant. The program comprises three steps, i.e., (i) the PDB file of the structures (7KQE), (ii) the alignment of the target sequence and recognized structures, and (iii) the visualization of the predicted structure using PyMol (http://www.pymol.org/). The Qualitative Model Energy ANalysis (QMEAN) and Global Model Quality Estimation (GMQE) values of the SWISS-MODEL server were used for assessing the fidelity of the structure. PROCHECK determines the stereochemical quality of the protein structure (http://www.ebi.ac.uk/thornton-srv/software/PROCHECK) [28] and was thus used for determining the attributes of the predicted 3D structure of SARS-CoV-2 B.1.617.1 variant S protein (QUX03874.1). Further, RAMPAGE was used to decipher the Ramachandran plot analysis of the model, which revealed the phi versus psi dihedral angles for each residue in the input PDB file, and also exhibited the allowed and disallowed regions for the in silico structured model based on the density-dependent smoothing.

RETRACTED

## 3. Results

### 3.1. Physicochemical Properties of the Proteins

The physicochemical properties of the protein QUX03874.1 of SARS-CoV-2 B.1.617.1 variant S protein were determined, which comprise 167 amino acids, and its molecular weight, total number of atoms, pI, and net charge are presented in Table 1. For QUX03874.1, the GRAVY index was -0.458, which indicated their hydrophilic nature. The II value of 14.45 for QUX03874.1, suggested the stability of this protein. Moreover, AI value of 65.33 for QUX03874.1 corroborated its stability over a wide range of temperature regime and consistent with earlier studies [29, 30].

### 3.2. Immunogenic Properties of SARS-CoV-2 B.1.617.1 Variant S Protein

The ABCpred and CTLpred were used for the determination of B-cell and T-cell epitopes for S protein of SARS-CoV-2 B.1.617.1 variant. Scores > 0.51 account for the potential epitope, and its higher probability. Therefore, the threshold value was set at 0.51 for a putative antigen. For the SARS-CoV-2 B.1.617.1 variant S protein, two potential B-cell and two T-cell linear epitopes revealed scores ≥ the threshold value of 0.8, which suggested their high propensity of being recognized (Table 2). B-cell epitope predictions showed 12 sequences having probability to be as epitope with score > 0.51. Among these, two peptide sequences TEIYQAGSTPCNGVQG and LQSYGFQPTNGVGYQP peptides at 60 and 82 positions were highly antigenic with scores 0.93 and 0.9, respectively. T-cell epitope predictions displayed 46 sequences as probable CTL epitope with score > 0.51. Among these, two peptides' sequences FERDISTEI and YRVVVLSFE at 54 and 98 positions with a highly antigenic score of 1 and 0.99, respectively. Further, QUX03874.1 of SARS-CoV-2 S protein displayed antigenic response with a score 0.56 and no IFN-*γ* response as predicted using the VaxiJen v2.0 and IFNepitope tool, respectively.

RETRACTED

### 3.3. In Silico Molecular Modeling of QUX03874.1 Coding Sequences of SARS-CoV-2 B.1.617.1 Variant S Protein

The sequence alignment of QUX03874.1 with the known structure 7KQE indicated that apart from the high % sequence identity (Table 3), some of the residues marked as stars are different from the known structure (Figure 1). The predicted topology showed that QUX03874.1 protein comprises two helices and five beta sheets (Figure 2). For the subsequent analysis, 7KQE was used as a reference for modeling the QUX03874.1 protein based on the already recognized electron microscopic structure of Homo sapiens viral protein (Human SARS coronavirus). The model generated was accurate for the angle and length of the bonds. SWISS-MODEL was then employed for generating a single model from the ClustalX files generated through sequence alignment and visualized qualitatively and quantitatively, which revealed the lowest root mean square deviation (RMSD) value with the template (Table 3; Figures 3(a) and 3(b)). Subsequently, the PROCHECK was employed for deciphering the stereochemistry (psi and phi angles) of the models, which produced several files comprising detailed data of the amino acids and the stringency of the generated structure (Table 4; Figure 4) in concurrence with the structures of the similar resolution [31]. The Ramachandran plot analysis of the recognized structures of QUX03874.1 revealed 84.2% of amino acids are in the most favored regions and 15.8% in additionally allowed regions, and no amino acid detected in the generously allowed and disallowed regions. Overall, the analysis revealed the fidelity of the predicted model and concurred with the 7KQE.

## 4. Discussion

The COVID-19 pandemic has resulted in a loss of more than 4 million human life with maximum casualties in the USA, Brazil, India, Mexico, Peru, Russian Federation, the UK, and Italy (as of September 16, 2021; https://www.worldometers.info/coronavirus/#countries). Further on, mutations and emergence of new variants of SARS-CoV-2 led to the surge of the second and third waves of COVID-19, and it has cost many lives. Among the different variants, B.1.617.1 has rapidly spread in India and to several countries throughout the world. Recent report has suggested that this variant is 6.8-fold less susceptible to neutralization by sera from COVID-19 convalescent and Moderna- and Pfizer-vaccinated individuals [32].

The number of deaths continues to increase across the globe, and there seems to be no respite from this menace. Therefore, there has been an unprecedented global endeavor almost at the war footing by the researchers to design and develop a potent vaccine against SARS-COV-2 B.1.617.1 variant to mitigate highly contagious and life-threatening COVID-19. In this context, an in silico approach for deciphering the structure and function of the S protein of SARS-CoV-2 B.1.617.1 variant is a pivotal prelude to the development of a potent vaccine.

RETRACTED

In the current paper, we have predicted the structure and functions of SARS-CoV-2 B.1.617.1 variant partial S protein using state of art bioinformatics approach. The validity of the predicted structure was also studied. Further, immunogenic properties of B.1.617.1 variant S protein using B-cell epitopes, T-cell epitopes, chemokines, antigen, and IFN-*γ* response prediction tools were also employed.

The 3D structures of some of the important proteins of SARS-CoV-2 have now been predicted [33–36; https://www.rcsb.org/]. Here, various physicochemical properties of the protein QUX03874.1 of B.1.617.1 variant S protein were deciphered. The high II values of protein (Table 1) and its hydrophilic nature suggested its high stability and thus deemed to be a potential candidate for engineering vaccine against COVID-19. The specific residues present in the protein act as antigenic epitopes [19].

*In silico* tool ABCpred, CTLpred, CHEMOpred, and Vaxijen servers were used for predicting the immunogenic properties of B.1.617.1 variant S protein (Table 2). Two potential B-cell linear epitopes were predicted with scores equal or more than 0.8 in QUX03874.1. This is in agreement with the recent study where B-cell epitopes have been predicted using Bepipred 2.0 [13, 37]. We also predicted and analyzed T cell epitopes in B.1.617.1 variant S protein. We found two potential T-cell epitopes with scores equal or above 0.99 in QUX03874.1. Hence, upon SARS-CoV-2 infection, both the arms of adaptive immunity (B and T cells) are likely to elicit immunological responses. The predicted immunoepitopes may play an important role in the initiation of the immune response.

The topology of the B.1.617.1 variant S protein revealed the fold comprising *α*-helices and *β*-sheets (Figure 2). It is the most prominent protein structure spanning the plasma membrane and can form hydrogen bonds, which confers stability [38]. Superimposition of QUX03874.1 with 7KQE revealed a high degree of structural overlap and sequence similarity, which was corroborated with the lowest RMSD (Table 3; Figures 3(a) and 3(b)). An earlier study has also reported an inverse correlation between the high incidence of the structural and sequence identity and RMSD value [39]. The QMEAN, *Z*-score, and analysis of the Ramachandran plot validated the high-quality of the 3D structure of QUX03874.1 (Table 4; Figure 4) and concurred with an earlier study on the hypothetical protein MG_377 in *Mycoplasma genitalium* [41]. The predicted model of QUX03874.1 could be used as a template for identifying the interaction of the protein and docking with the ligand and putative drugs, which may aid in the discovery of novel drug molecules for fighting the viral disease. However, at present, the function of QUX03874.1 remains enigmatic and merits in-depth studies involving their three-dimensional X-ray structural analysis and posttranslational modifications.

RETRACTED

## 5. Conclusion

An in silico approach was employed for deciphering the structure and key immunogenic properties, for partial S protein of SARS-CoV-2 B.1.617.1 variant. The study provides valuable insights that could be useful for the development of monoclonal antibodies, inhibitors, or vaccines targeting S protein of SARS-CoV-2 B.1.617.1 variant, as well as diagnostic tools shortly, which warrants empirical validation by rigorous and stringent wet-lab experiments.

## Figures and Tables

**Figure 1:** Sequence alignment of QUX03874.1 protein with the 7KQE from *Homo sapiens* viral protein: the amino acids that differ in the alignment were highlighted with blue color.

**Figure 2:** Topology diagram of S protein showing the overall fold: *α*-helices are indicated by red cylinders and *β*-sheets by pink arrow.

**Figure 3:** Homology modeling and superposition of the structures from QUX03874.1 protein. (a) Modeled structure of QUX03874.1 represented as cyan color and N and C terminal marked. (b) Superposition of QUX03874.1 with the template 7KQE represented as cyan and purple in color, respectively.

**Figure 4:** Ramachandran plot generated by PROCHECK software show Psi and Phi bond angles, white regions coincide to sterically disallowed region, red areas coincide to allowed regions, and yellow regions correspond to the atoms in the generously allowed regions for QUX03874.1.

**Table 1:** Physiochemical properties of the QUX03874.1 S protein from SARS-CoV-2 computed using ExPASy ProtParam tool.

No.	Properties	QUX03874.1
1.	Number of amino acids	167
2.	Molecular weight (kDa)	18.608
3.	Formula	C_837_H_1268_N_226_O_247_S_5_
4.	Total number of atoms	2583
5.	Theoretical pI	9.09
6.	EC	20650
7.	AI	65.33
8.	GRAVY	-0.458 (hydrophilic)
9.	II	14.45 (protein is stable)

**Table 2:** Prediction of epitopes (B and CTL), IFN-*γ* response, and probable antigen of SARS-CoV-2 B.1.617.1 variant S protein (QUX03874.1).

B-cell epitope				CTL epitope				Antigen potential	Chemokine
Rank	Position	Sequences/IFN-*γ* response	Score	Rank	Position	Sequences/IFN-*γ* response	Score	Prediction score	Prediction
1	60	TEIYQAGSTPCNGVQG/negative	0.93	1	54	FERDISTEI/negative	1.00	0.5656	Nonchemokine
2	82	LQSYGFQPTNGVGYQP/negative	0.90	2	98	YRVVVLSFE/negative	0.99		Nonchemokine

RETRACTED

**Table 3:** Sequence identity between the template and the modeled structure.

Modeled structure	Most favored regions	Additional allowed regions	Generously allowed regions	Disallowed regions
QUX03874.1	84.2%	15.8%	0.0%	0.0%

**Table 4:** Ramachandran plot statistics of modeled structure of the QUX03874.1 S protein from SARS-CoV-2 B.1.617.1 variant.

Accession number	Template	Sequence identity (%)	RMSD deviation (Å)
QUX03874.1	7KQE	98.8	0.23

## Data Availability

All the data in this manuscript is available with the corresponding author upon formal request.
